RETRACTED

# Mechanism of Hepatoprotective Effect of *Boesenbergia rotunda* in Thioacetamide-Induced Liver Damage in Rats

**DOI:** 10.1155/2013/157456

**Published:** 2013-08-07

**Authors:** Suzy M. Salama, Mahmood A. Abdulla, Ahmed S. AlRashdi, A. Hamid A. Hadi

**Affiliations:** ^1^Department of Biomedical Science, Faculty of Medicine, University of Malaya, 50603 Kuala Lumpur, Malaysia; ^2^Department of Chemistry, Faculty of Science, University of Malaya, 50603 Kuala Lumpur, Malaysia

## Abstract

*Background*. Researchers focused on developing traditional therapies as pharmacological medicines to treat liver cirrhosis. *Objectives*. Evaluating the hepatoprotective activity of *Boesenbergia rotunda* (BR) rhizome ethanolic extract on thioacetamide-induced liver cirrhosis in rats. *Methods*. Male *Sprague-Dawley *rats were intraperitoneally injected with 200 mg/kg TAA 3 times/week and daily oral administration of 250 mg/kg, 500 mg/kg of BR extract, and 50 mg/kg of the reference drug Silymarin for 8 weeks. At the end of the experiment, Masson's trichrome staining was used to measure the degree of liver fibrosis. Hepatic antioxidant enzymes (CAT and GPx), nitrotyrosine, cytochrome (P450 2E1), matrix metalloproteinase (MMP-2 and MMP-9), tissue inhibitor of metalloproteinase (TIMP-1), and urinary 8-hydroxyguanosine were measured. Serum levels of transforming growth factor TGF-**β**1, nuclear transcription factor NF-**κ**B, proinflammatory cytokine IL-6, and caspase-3 were evaluated. Serum protein expression and immunohistochemistry of proapoptotic Bax and antiapoptotic Bcl-2 proteins were measured and confirmed by immunohistochemistry of Bax, Bcl-2, and proliferating cell nuclear antigen (PCNA). *Results*. BR treatment improved liver histopathology, immunohistochemistry, and biochemistry, triggered apoptosis, and inhibited cytokines, extracellular matrix proteins, and hepatocytes proliferation. *Conclusion*. Liver cirrhosis progression can be inhibited by the antioxidant and anti-inflammatory activities of BR ethanolic extract while preserving the normal liver status.

## 1. Introduction

Pharmaceutical drugs that depend on compounds such as colchicine and interferons are currently available for the treatment of liver cirrhosis but with either unreliable efficacies or high situations of side effects [1]. A number of natural compounds produced from vegetation offer alternative healthcare options that are more effective and safe [2]. Ingredients from recently found or already known plant varieties are regularly being examined on experimental animals [3]. The prospective tasks and efficiency of plant extracts in liver diseases are yet to be analyzed. The ethanolic extract of *Curcuma longa *rhizomes extract was recently proved to exhibit hepatoprotective efficacy against TAA intoxication in rats [4]. A large number of medicinal plants with hepatoprotective activity have been reported by several researchers [5, 6].* Boesenbergia rotunda* (BR) rhizomes is one that is awaiting more analysis of its part in the pathology of the liver.

RETRACTED

*Boesenbergia rotunda* is one of the species that belongs to family Zingiberaceae and is traditionally used in folk medicine in Southeast Asia and commonly known as temu kunci. Medical research in the past used different solvents in preparing extracts from BR such as methanol, chloroform, and hexane. The methanol extract of BR was found to contain Quercetin and Kaempferol, which are well-known antioxidant and anti-inflammatory [7]. Chloroform or hexane extract of BR was found to contain other important flavanones and chalcones which are highly antioxidant compounds [8]. Furthermore, previous studies have revealed various bioactivities of BR rhizome extract such as anticancer [9], antibacterial [10], wound healing activity [11], and antiulcerogenic [12]. Our previous study examined the effectiveness of the ethanol-based extract of BR as a preventive therapy on a rat model of liver cirrhosis induced by thioacetamide, and our results revealed that BR extract exhibited significant hepatoprotective activity [13]. As an extension of our initiatives, in this study, we studied the mechanism of the protective effect of BR ethanol extract in TAA intoxication. Silymarin was also used in our study as a well-known hepatoprotectant reference drug extracted from the seeds of *Silybum marinum* plant [14].

## 2. Materials and Methods

### 2.1. Animals

Thirty male *Sprague-Dawley* rats (180–250 g) were used in the study. The rats were held in cages with wire bottoms at 25 ± 2°C, given tap water and conventional pellet, and revealed to a 12 hours of light-dark cycle at 50–60% moisture in well-prepared animal house. Throughout the test, all animals obtained individual proper care according to the requirements defined in the “Guide for the Care and Use of Laboratory Animals” readified by the Nationwide Academia of Sciences and released by the National Institution of Health. The research was accepted by the Committee Panel for Animal Analysis, Faculty of Medicine, University of Malaya, Malaysia PM/28/08/2009/MAA.

### 2.2. Experiment

Animal groups were divided into 5 categories of 6 rats each (Table 1). TAA was ready by complete dissolving of TAA crystals (Sigma-Aldrich, USA) in sterile distilled water [15]. Silymarin (International Clinical, USA) was used as a reference drug and prepared by complete dissolving in 10% Tween-20.

RETRACTED

At the end of the experimental period, the rats were sacrificed, and blood was collected as mentioned in our previous work [13]. Liver tissues were excised, cleaned with ice-cold normal saline, and blotted, and some tissues were prepared for histopathology and immunohistochemistry evaluation. Some other liver tissues were washed in 0.02 mol/L PBS (pH 7.0–7.2) to get rid of excess blood. One gram of each liver was sampled and homogenized (10% w/v) in 50 mM cold potassium phosphate buffer (pH 7.4) by using teflon homogenizer (Polytron, Heidolph RZR 1, Germany). The resulting tissue homogenate was allowed to centrifuge at 3500 rpm for 10 minutes at 4°C in a centrifuge (Heraeus, Germany). The collected supernatant was divided into aliquots and then kept at −80°C till being assayed. The protein content in the liver tissue homogenate collected from all animals was assayed by using bovine serum albumen (BSA) according to Lowry method [16]. Blood samples were collected from all rats into carefully labeled tubes containing activated gel and allowed to clot and centrifuge at 3000 rpm for 10 min at 4°C. The collected serum samples were divided into aliquots and then kept at −80°C. Clean urine samples from all animals were collected 24 hours before sacrifice and kept at −80°C before assaying for levels of 8-hydroxy-deoxyguanosine.

### 2.3. Liver Tissue Content of CYP2E1

The cytochrome enzyme (CYP2E1) plays a crucial role in the metabolism of TAA in the liver microsome [17]. Aliquots of the tissue homogenate from all rats were tested for the level of CYP2E1 enzyme using microtiter plate precoated with monoclonal antibody specific to rat CYP2E1 and following the instructions of Uscn Life Science sandwich enzyme immunoassay (E90988Ra, China).

### 2.4. Evaluation of Urine 8-OH-dG and Hepatic Nitrotyrosine

The free radicals generated from biotransformation of TAA in the liver result in oxidative damage via their covalent binding to the macromolecules of hepatocytes including DNA, protein, and lipid molecules causing necrosis of hepatocytes [18]. In our previous study, the level of malondialdehyde has been evaluated in the liver tissue homogenate [13]. In this study, the hepatic level of nitrotyrosine was measured as a marker for protein oxidation [19] utilizing a multiclonal anti-nitrotyrosine antibody and nitrotyrosine-horseradish conjugate as per the company's manuals (MyBiosource MBS722419, USA). Urine level of 8-hydroxy-deoxyguanosine (8-OH-dG) was evaluated as a marker for DNA oxidation [20] using monoclonal antibody specific to 8-OH-dG and following the kit instructions (Genox KOG-HS10E, USA). The principle of the assay is based on a competitive enzyme-linked immunoabsorbent method for measuring the quantity of 8-hydroxy-2′-deoxyguanosine adduct resulting from DNA oxidation.

RETRACTED

### 2.5. Evaluation of Antioxidant Enzymes (CAT and GPx)

Endogenous antioxidants, SOD, CAT, and GPx signify the first array of protection against the harms of free radicals and are essential for avoiding or at least reducing the occurrence and development of diseases [21]. In our previous experiment, we evaluated the level of superoxide dismutase (SOD) in the liver tissue homogenate of rats. In this study, the levels of catalase (CAT) and glutathione peroxidase (GPx) enzymes were assayed in the liver tissue homogenate collected from all animals following the instructions of Cayman kits (Sigma Cat no. 707002 and no. 703102, resp.). In brief, CAT activity was evaluated by Purpald Chromagen measuring the formaldehyde produced by the reaction of CAT enzyme with methanol in the presence of H_2_O_2_. The principle of GPx assay depends on the indirect measure of GPx activity by a coupled reaction. GPx reduces hydroperoxide into the oxidized form glutathione (GSSG) which is recycled by NADPH into its reduced form glutathione reductase (GR). All assays were performed in triplicate.

### 2.6. Assessment of Cytokines and Chemokines

Sera aliquots collected from all rats were assayed for transforming growth factor-beta (TGF-*β*1) as a fibrogenesis-driving cytokine [22] using an ELISA microtiter plate precoated with rat TGF-*β*1 specific-specific polyclonal antibodies as per the manufacturers' instructions (Abnova, KA0416, USA). The nuclear transcription factor NF-*κ*B and the proinflammatory cytokine interleukin IL-6 as important signals in liver injury [23] were assayed by enzyme-linked immunosorbent assay using ELISA microtiter plates precoated with antibodies specific to NF-*κ*B or IL-6 according to the instructions of the manufacturer (Uscn Life Science E91824Ra, China, for NF-*κ*B and E90079Ra for IL-6).

### 2.7. Assessment of Caspase-3, Proapoptotic Bax, and Antiapoptotic Bcl-2

Based on many studies, it was found that the triad Bax, Bcl-2, and caspase-3 are involved in the apoptosis of hepatocytes during liver injury [24]. To demonstrate the effect of BR rhizome extract on the apoptosis of liver cells, rat Bax ELISA kit (Uscn Life Science E91824Ra, China), rat Bcl-2 ELISA kit (Uscn Life Science E90778Ra, China), and rat caspase-3 ELISA kit (Uscn Life Science E90626Ra, China) were applied utilizing 96-well plates precoated with monoclonal antibody specific to Bax, Bcl-2, or caspase-3 for the evaluation of the levels of Bax, Bcl-2, and caspase-3 respectively, in the sera aliquots collected from all rats. 

### 2.8. Evaluation of Matrix Metalloproteinase Enzymes (MMP-2 and MMP-9) and TIMP-1

Matrix metalloproteinase enzymes (MMP-2 and MMP-9) and their partial regulator tissue inhibitor of metalloproteinase (TIMP-1) play a role in liver damage [25]. For this purpose, tissue homogenates were assayed for the level of these markers by monoclonal antibodies specific to the tested antigen following the kits' manuals (Uscn Life Science E90100Ra, E90553Ra, and E90552Ra, China).

RETRACTED

### 2.9. Histopathological Analysis

Five *μ*m thick sections of liver samples were prepared for Masson's trichrome (Sigma, USA) staining as a marker for detecting the degree of fibrosis [26] and observing the collagen fibers developed in liver tissues [27]. Examination of the slides was performed under a light microscope, and digital images were captured using a Nikon microscope (Y-THS, Japan) (magnification ×20).

### 2.10. Immunohistochemistry

Using poly-L-lysine-coated slides, liver sections were prepared and heated in an oven (Venticell, MMM, Einrichtungen, Germany) for 25 minutes at 60°C. After heating, liver sections were deparaffinized in xylene and rehydrated in graded alcohol. Sodium citrate buffer of concentration 10 mM was heated till boiling in a microwave for antigen retrieval. Immunohistochemistry staining was applied following the manual of the company (DakoCytomation, USA). Succinctly, 0.03% hydrogen peroxide sodium azide was used to block the endogenous peroxidase for 5 min followed by washing the tissue sections carefully using wash buffer and then incubated with Bcl-2-associated X protein (Bax) (1 : 500), proliferating cell nuclear antigen (PCNA) (1 : 200), and antiapoptotic protein Bcl-2 (1 : 50) (Santa Cruz Biotechnology Inc., California, USA) biotinylated primary antibodies for 15 minutes. After incubation, tissue sections were carefully rewashed with washing buffer and conserved in the buffer bath. After adding streptavidin-HRP, sections were kept for 15 minutes incubated and then washed. Diaminobenzidine substrate chromagen was applied to the sections and reincubated for over 8 min followed by careful washes and hematoxylin counterstaining for 5 seconds. Weak ammonia (0.037 mol/L) was used for dipping the sections 10 times and then washed and cover slipped. Light microscopy was used to examine the brown-stained positive antigens.

### 2.11. Statistical Analysis

Statistical analysis of the results was performed using one-way ANOVA followed by Tukey post hoc test analysis using SPSS (Version 18, SPSS Inc., Chicago, IL, USA). A value of *P* < 0.05 was considered statistically significant between the measurements of the two compared groups. All values were reported as mean ± SEM.

RETRACTED

## 3. Results

### 3.1. Hepatic Level of CYP2E1

The result of the effect of BR extract on the hepatic cytochrome enzyme CYP2E1 is shown in Figure 1. Animals from cirrhosis group had significantly (*P* < 0.01) higher levels (2.85 ± 0.12 ng/mL) of CYP2E1 compared with normal group (0.96 ± 0.36 ng/mL) and reference group (1.14 ± 0.05 ng/mL). Low dose and high dose BR-treated rats showed significantly (*P* < 0.01) lower levels (1.37 ± 0.15 and 1.10 ± 0.09 ng/mL, resp.) when compared with cirrhosis group. 

### 3.2. Level of Oxidative Stress

Oxidative stress markers (hepatic nitrotyrosine and urinary 8-OH-dG) are shown in Table 2. Generally, cirrhosis rats had significantly higher levels of oxidative stress parameters (*P* < 0.001) than normal rats and the treated groups. Remarkably, low dose and high dose-BR treated rats showed significantly lower levels (*P* < 0.001) of liver nitrotyrosine and urinary 8-OH-dG compared to cirrhosis group. Moreover, no significant differences were observed in the tested oxidative stress parameters between the animals treated with the plant extract and those treated with silymarin. These results suggest that BR treatment may protect liver tissues from progressive damage during liver injury.

### 3.3. Hepatocellular Endogenous Enzymes

Hepatocytes loss in the cirrhotic livers of rats was analyzed in another way by the activity of antioxidant enzymes CAT and GPx and the results are shown in Table 3. CAT and GPx, results were similar to that of the oxidative stress parameters but in the opposite manner, so the values of CAT and GPx in the rats of the cirrhosis group were lower than that in normal rats. These results revealed the occurrence of extensively injured hepatocytes of cirrhotic livers. Daily oral administration of low and high dose BR extract significantly (*P* < 0.01) increased the levels of CAT and GPx and induced the survival of hepatocytes. These results conjointly with our previous results of SOD [13] support the approach that treatment with BR extract could provide a healthy status for protecting the hepatic cells from advanced damage.

### 3.4. Cytokines and Chemokines Assessment

The serum levels of TGF-*β*1, NF-*κ*B, and IL-6 from the samples collected from all sacrificed rats are shown in Figure 2. Results showed that the serum levels of TGF-*β*1, NF-*κ*B, and IL-6 were significantly elevated (*P* < 0.05) in the samples from cirrhosis group (100.00 ± 10.00 pg/mL, 2.86 ± 0.06 ng/mL and 288.58 ± 11.15 pg/mL, resp.) compared to the other animal groups. Administration of BR extract to animals attenuated the levels of the fibrogenesis agent TGF-*β*1 to 81.67 ± 1.67 pg/mL and the inflammatory mediators NF-*κ*B and IL-6 to 1.93 ± 0.05 ng/mL and 148.12 ± 15.61 pg/mL, respectively, in the low dose BR-treated rats and 58.33 ± 4.41 pg/mL, 1.43 ± 0.07 ng/mL and 129.50 ± 3.79 pg/mL, respectively, in the high dose BR-treated rats. Levels of TGF-*β*1, NF-*κ*B, and IL-6 from the high dose BR-treated group approached the values obtained from the reference group Silymarin (63.33 ± 1.67 pg/mL, 1.49 ± 0.06 ng/mL, and 125.35 ± 5.06 pg/mL, resp.) compared to the higher value in the low dose BR-treated group. Results suggest that BR extract has dose-dependent nature in its inhibitory effect to the profibrogenic and proinflammatory cytokines and NF-*κ*B chemokine.

RETRACTED

### 3.5. Serum Level of Caspase-3, Bax, and Bcl-2

The levels of the proapoptotic protein Bax and the antiapoptotic protein Bcl-2 in the rat sera are shown in Figure 3(a), and the ratio of Bax/Bcl-2 is shown in Figure 3(b). Bax results showed no significance between cirrhosis and normal group rats (1.61 ± 0.15 and 1.07 ± 0.04 ng/mL resp.). On the other hand, there was significant increase (*P* < 0.05) in the level of Bax from reference and high dose BR-treated groups (4.95 ± 0.11 and 4.68 ± 0.19 ng/mL, resp.) compared to cirrhosis group. On the contrary, the level of antiapoptotic protein Bcl-2 showed significant increase (*P* < 0.05) in the cirrhosis group compared to normal group (2.57 ± 0.23 and 0.89 ± 0.09 ng/mL, resp.), whereas no significance observed between any of the treated groups when compared with cirrhosis group indicating enhanced apoptosis in silymarin and BR*-*treated groups as confirmed by the ratio Bax/Bcl-2 in Figure 3(b). Furthermore, the serum level of caspase-3 in the cirrhosis group was not significantly higher (2.11 ± 0.48 ng/mL) compared to normal group (1.43 ± 0.33 ng/mL) as illustrated in Figure 3(c). Treating the cirrhotic livers with silymarin or high dose BR elevated the caspase-3 value to reach 5.54 ± 0.27 and 5.83 ± 0.19 ng/mL, respectively. The similarity observed in the results of Bax and caspase-3 confirms the enhancement of apoptosis by BR extract in the same manner as the reference drug, silymarin.  Figure 3(d) shows the relation between Bax, Bcl-2, and caspase-3 in all the experimental groups. Results showed parallel increase in the serum level of Bax and caspase-3 in silymarin and BR groups, whereas Bcl-2 level showed reversed serum level suggesting increased apoptosis in the treated groups compared to cirrhosis control group.

### 3.6. Hepatic TIMP-1, MMP-9, and MMP-2

The results of the effect of BR extract treatment on the liver tissue homogenate level of MMP-2, MMP-9, and TIMP-1 collected from all experimental animals are illustrated in Table 4. From the results, the level of the tested enzymes were significantly high (*P* < 0.05) in the cirrhosis group rats compared to all other groups. On the other hand, administration of BR extract to the animals significantly (*P* < 0.05) attenuated the enzymatic levels of MMP-2, MMP-9, and TIMP-1 to approach the values of the reference control group with the exception of the low dose BR-treated group which did not show significance to cirrhosis group indicating the efficacy of the plant extract treatment in a dose-dependent manner. Results in Table 4 showed parallel decrease in the hepatic level of MMP-2, MMP-9, and TIMP-1 from BR-treated groups.

RETRACTED

### 3.7. Masson's Trichrome Staining

The degree of fibrosis determined by Masson's trichrome staining of the liver sections from all the treated groups is shown in Figure 4. Liver sections from normal rats appeared normal without signs of collagen deposition. Liver sections from the cirrhosis rats of cirrhosis group revealed increased deposition of collagen fibers around the congested central vein indicating severe fibrosis. Liver tissues from the reference group showed minimal collagen deposition indicating minimal fibrosis. Livers from rats treated with low dose BR extract showed moderate deposition of collagen fibers and moderate congestion around the central vein, while those from rats treated with high dose BR extract showed mild collagen deposition and mild congestion around the central vein. This measurement of the degree of fibrosis confirms the previous findings that treatment with BR extract might protect the animals' liver from development of fibrosis.

### 3.8. Immunohistochemistry

Bax, Bcl-2, and PCNA staining of liver cells from all animal groups are shown in Figures 5(a), 5(b), and 6. Hepatocytes of liver tissues from cirrhosis group rats showed downregulation of Bax staining with upregulation of Bcl-2-positive hepatocytes and more PCNA staining indicating severe necrosis with high cell proliferation to repair the damaged hepatocytes. Hepatocytes from the reference group (Silymarin-treated rats) showed upregulated Bax expression, downregulated Bcl-2 expression, and few PCNA staining indicating lower levels of proliferation of necrotized hepatocytes proliferation than apoptosis. Liver tissues treated with low dose and high dose BR extract induced hepatocyte apoptosis as indicated by the upregulated Bax expression, downregulated Bcl-2, and downregulated proliferation of necrotic hepatocytes as indicated by reduced PCNA staining. These findings support the idea of BR extract-induced hepatoprotective activities against progressive liver damage by increasing apoptosis of damaged hepatocytes and ameliorating their proliferation.

RETRACTED

## 4. Discussion

Liver cirrhosis has become a serious health problem because of the wider use of prescribed medications with adverse reactions in modern life of today or the drug misuse. Consequently, the current research has targeted on finding new therapeutic alternatives and analyzing their mechanism to get rid of the signaling routes and reduce the loss induced on the liver [28]. Beyond the techniques with artificial pharmacology, the search also chases alternative techniques that depend on natural products. In particular, it targets those plants with known medical history or confirmed prospective of positive results against the illnesses of the liver or other body parts [29]. To aid these initiatives, in this study, we analyzed the mechanism of ethanol extract of BR rhizomes as a promising therapy for treating liver cirrhosis.

Thioacetamide is biotransformed by CYP2E1 enzymes located in the microsomes of liver cells and convert it to a highly reactive toxic intermediate known as thioacetamide sulphur dioxide through oxidation [30], inducing hepatotoxicity in experimental animals and different grades of liver damage including nodular cirrhosis, production of pseudolobules, proliferation of hepatic cells, and necrosis of parenchyma cells [31]. All experimental animals in the present study were tested for CYP2E1 enzyme level in liver homogenate tissues (Figure 1). Efficacy of BR extract in comparison with silymarin control was able to inhibit metabolism of TAA, which might be one of the significant factors in hepatoprotective activity by blocking the release of toxic metabolites and ROS responsible for inducing damage of hepatocytes [32].

Reactive oxygen species (ROS) and reactive nitrogen species (RNS) production increase during liver injury by transformation of xenobiotics such as CCl_4_, ethanol, and acetaminophen in the liver and play a crucial role in the death of hepatocytes [33]. TAA induces hepatocyte damage via its metabolite, TASO_2_, which damages the macromolecules of hepatocytes causing damage of DNA molecules, oxidation of protein molecules, and peroxidation of the cell membrane biomolecules [34, 35]. This study evaluated the oxidative stress markers and observed the degree of liver cells damage. The levels of urine 8-OH-dG and nitrotyrosine (Table 2) were high in the cirrhosis group compared to the treated groups. This supported the crude extract antioxidants mechanism in downregulating ROS, inhibiting DNA damage, and attenuating protein and lipid oxidation [36]. Furthermore, the antioxidant constituents of BR extract helped in boosting the hepatocellular endogenous enzymes (CAT and GPx) as shown in Table 3.

Toxins target metabolically effective hepatic cells causing dysfunction of hepatocytes and the discharge of inflammation-related cytokines as NF-*κ*B and IL-6 and fibrogenic mediators as TGF-*β*1. Many researchers have recommended that part of liver injury brought on by TAA is mediated through oxidative stress and the effect of cytokines via fat peroxidation [37, 38]. The free radicals released as the consequences of TAA metabolism in liver cells activate myofibroblasts that secrete fibrinogen and growth factors [39]. The present study revealed that BR extract treatment attenuated level of the prominent profibrogenic cytokine TGF-*β*1 (Figure 2) indicating the inhibitory activity of BR extract to the proliferative activity of HSCs which might be confirmed by the less collagen deposition in the liver tissues of animals treated with BR extract (Figure 4). Similarly, the high levels of proinflammatory cytokines IL-6 and NF-*κ*B (Figure 2) observed in the cirrhosis group rats were reversed in the rats treated with BR extract indicating the anti-inflammatory activity of BR extract.

RETRACTED

A number of studies have focused on the molecular regulation of apoptosis. One of the characteristic features of liver diseases is the death of hepatocytes as a response to drug/toxicant-induced liver injury. Cytotoxic drugs and cellular stress activate the intrinsic mitochondrial apoptotic pathway [40] so that the inhibitors of Bcl-2 activate caspase-3 initiating apoptosis, whereas inducers of Bcl-2 induce necrosis of cells [41]. *In vivo*, necrotic death is often associated with extensive damage in the tissue resulting in necro-inflammatory response [42]. Although toxicity induced by TAA was reported to cause upregulation of Bax protein and downregulation of the antiapoptotic protein Bcl-2 and its translocation into the mitochondria, causing apoptosis [43] but other studies suggested that the ROS produced from thioacetamide biotransformation causes centrolobular necrosis [44]. Some Plant extracts such as *Curcuma longa* extract [4] and some antioxidants such as *α*-lipoic acid [45], curcumin, and curcuminoids [46] were proved to induce apoptosis. In the current study, we observed significant increase in the serum level of Bax protein and caspase-3 and decrease in Bcl-2 protein in the BR-treated and silymarin-treated animals compared to cirrhosis group animals as shown in the relation between Bax, Bcl-2, and caspase-3 in Figure 3(d). This was confirmed by the ratio Bax/Bcl-2 (Figure 3(b)) which was high in the treated groups compared to cirrhosis group and the immunohistochemistry staining of Bax and Bcl-2 (Figure 5). The ethanolic extract of BR rhizomes might contain active compounds such as the chalcone Boesenbergin A [47] and the sesquiterpene zerumbone [48] which were reported recently to induce apoptosis of liver cancer cells HepG2 through the release of cytochrome C and the formation of caspase-3 modifying the necrotic effect due to TAA intoxication to apoptosis. This modification *in vivo* would scale down the release of inflammatory mediators that would prevent progressive liver damage. Furthermore, feeding of rats daily with BR extract along with TAA injections 3 times/week for 8 weeks inhibited proliferation of hepatocytes as indicated by the significant reduction of PCNA staining in the liver sections from the plant extracts-treated groups similar to that in the Silymarin-treated group (Figure 6) [49]. Downregulation of cell proliferation in BR-treated rats may be attributed to the reduced damage in the BR-treated livers compared to the higher damage of hepatocytes and the upregulation of PCNA in the cirrhosis animals to regenerate the necrotic effect of TAA to hepatocytes.

RETRACTED

In liver fibrosis, there is an imbalance between excess deposition and/or a decrease in the extracellular matrix (ECM) removal with consequent scarring damage [50]. ECM is mainly controlled by matrix metalloproteinases (MMPs), which are a group of proteolytic enzymes that are able to degrade the ECM [51, 52]. MMP-9 and TIMP-1 were verified as the molecular signatures during the progress of liver cirrhosis induced by TAA [53]. Park et al. observed that TAA increased MMP-2 expression in the liver tissues of rats and reported that the balance of MMPs and TIMPs is the key factor of liver fibrogenesis [50]. In this research, administered animals with plants extract showed significant downregulation in the hepatic level of TIMP-1, MMP-9 and MMP-2 similar to silymarin reference group (Table 4). Results suggest that the efficacy of BR extract might be due to the inhibition of HSCs and kupffer cells activity and their secretion to MMP-2 and MMP-9, respectively. In addition, reduced activity of HSCs as indicated by the decreased level of collagen deposition in the BR-treated liver tissues has led to down-regulation of TIMP-1 [54]. Furthermore, the reduced activity of kupffer cells was indicated by the significant inhibitory effect of BR extract to the mediators TGF-*β*1, IL-6, and NF-*κ*B levels in rat serum. Consequently, the low level of these mediators might have contributed to HSCs activation and reduced liver injury [19].  Figure 7 summarizes the effect of BR treatment on the liver damage induced by TAA intoxication.

Due to the crucial role played by HSCs in liver fibrosis via their resistance to apoptosis, recent treatment strategies of liver diseases are to inhibit their proliferation or induce their apoptosis. The biochemical findings of our study were confirmed by the histopathological examinations of rat liver tissues (Figure 4) showing that livers from BR-treated rats had nearly normal liver architecture with significant reduction in collagen synthesis. This was probably due to the inhibitory effect of the plant extract on hepatic stellate cell activation. Inhibition of HSC activation and downregulation of collagen-I in the livers treated with BR extract might be due to the activity of polyphenol constituents in BR extract [55].

RETRACTED

## Figures and Tables

**Figure 1:** Effect of *B. rotunda *(BR) extract on hepatic levels of cytochrome enzyme CYP2E1 in rats at the end of the experiment. Data were expressed as mean ± SEM. **P < 0.01 compared with the normal group. *P < 0.01 compared with cirrhosis group.

**Figure 2:** Effect of BR extract on the serum level of TGF-*β*1, NF-*κ*B, and IL-6 in rats at the end of the experiment. (a) TGF-*β*1, (b) NF-*κ*B, and (c) IL-6. Data were expressed as mean ± SEM. Means among groups (*n* = 6 rats/group) show significant difference. **P < 0.001 compared to the normal group. *P < 0.001 compared to cirrhosis group. ^#^ *P* < 0.01 compared to cirrhosis group.

**Figure 3:** Effect of BR extract on the serum level of (a) Bax and Bcl-2, (b) Bax/Bcl-2 ratio, (c) caspase-3, and (d) relation between Bax, Bcl-2, and caspase-3 at the end of the experiment. Data were expressed as mean ± SEM. *P < 0.05 compared with the cirrhosis group. **P < 0.05 compared to the normal group.

**Figure 4:** Masson's trichrome staining of representative livers sampled from rats in different experimental groups. (a) Normal liver did not show signs of collagen deposition in livers from a normal rat. (b) Severe collagen deposition (arrow) and severe fibrosis were seen in the livers from a cirrhosis rat. (c) Minor collagen deposition in the liver of a hepatoprotected rat treated with Silymarin. (d) Moderated collagen deposition and moderate congestion around the central vein in the liver of rats treated with low dose BR extract. (e) Mild collagen deposition was observed in the livers of rats treated with high dose BR extract (original magnification ×20).

**Figure 5:** Immunohistochemistry staining of (a) Bax and (b) Bcl-2 of representative livers sampled from rats in different experimental groups. Less apoptosis indicated by (ia) few Bax-positive hepatocytes (white arrow) and (ib) more Bcl-2-positive hepatocytes (black arrow) in liver tissues from a cirrhosis rat group. (iia) High numbers of Bax-positive hepatocytes (White arrow) and (iib) very less Bcl-2-positive hepatocytes (black arrow) in the liver from a hepatoprotected rat treated with Silymarin. Moderate apoptosis as indicated by (iiia) moderate Bax staining (white arrow) and (iiib) moderate Bcl-2 staining (black arrow) indicating moderate apoptosis in the liver from the rats treated with low dose BR extract. (iva) High numbers of Bax-positive cells (white arrow) with severe apoptosis and (ivb) very less Bcl-2-positive hepatocytes (black arrow) were observed in the liver of the rats treated with high dose BR extract (original magnification ×40).

RETRACTED

**Figure 6:** Immunohistochemistry staining of PCNA of livers sampled from rats in different experimental groups. (a) Normal livers did not show signs of PCNA expression in hepatocytes from control rats. (b) Cirrhosis control liver showed severe fibrosis with greater PCNA expression in the necrotized hepatocytes. (c) Silymarin-treated liver showed less PCNA-stained hepatocytes (arrow) indicating less hepatocyte proliferation. (d) The low dose BR-treated liver showed moderate hepatocyte proliferation as indicated by moderate PCNA staining (arrow) in the hepatocytes. (e) High dose BR-treated livers showed minor PCNA expression (arrow) with few proliferated necrotized hepatocytes which were observed in the liver (original magnification ×40).

**Figure 7:** Possible mechanism of hepatoprotective effect of *Boesenbergia rotunda* on TAA-induced liver damage in rats.

**Table 1:** Experimental design.

Group	Number of animals	Intraperitoneal injection (three times/week)	Oral administration (5 mL/kg)	Durations (weeks)
Normal control	6	Sterile distilled water (1 mL/kg)	10% Tween-20	8
Cirrhosis control	6	TAA	10% Tween-20	8
Reference control	6	TAA	Silymarin 50 mg/kg	8
Low dose *B. rotunda *	6	TAA	*B. rotunda *250 mg/Kg	8
High dose *B. rotunda *	6	TAA	*B. rotunda* 500 mg/kg	8

**Table 2:** Effect of BR extract on urine OH-dG and liver tissue homogenate level of nitrotyrosine from the rats at the end of the experiment.

Group	8-OH-dG ng/mL	Nitrotyrosine (ng/mL)
Normal group	2.17 ± 0.33	1.06 ± 0.07
Cirrhosis group	5.40 ± 0.34**	3.87 ± 0.13**
Reference group	2.80 ± 0.15*	1.67 ± 0.07*
Low dose BR	2.83 ± 0.33*	1.40 ± 0.20*
High dose BR	2.37 ± 0.88*	1.33 ± 0.13*

8-OH-DG; 8-hydroxy-deoxyguanosine. Data are expressed as mean ± SEM. Means among groups (*n* = 6 rats/group) show significant difference. *P < 0.001 compared with cirrhosis group. **P < 0.001 compared with normal group.

**Table 3:** Effect of BR extract on the liver tissue homogenate level of CAT and GPx from the rats at the end of the experiment.

Group	CAT (nmoL/min/mg protein)	GPx (nmoL/min/mg protein)
Normal control	54.00 ± 0.36	860.37 ± 19.32
Cirrhosis control	27.49 ± 1.67**	451.00 ± 89.68^##^
Reference control	52.76 ± 3.29*	926.11 ± 36.42*
Low dose BR	41.34 ± 2.74^#^	902.59 ± 69.09^#^
High dose BR	51.42 ± 1.34*	975.05 ± 54.08*

CAT: catalase, GPx: glutathione peroxidase. Data are expressed as mean ± SEM. Means among groups (*n* = 6 rats/group) show significant difference. *P < 0.001 compared with cirrhosis group. **P < 0.001 compared with normal group. ^#^ *P* < 0.01 compared with cirrhosis group. ^##^ *P* < 0.01 compared with normal group.

RETRACTED

**Table 4:** Effect of BR extract on the liver tissue homogenate level of MMP-2, MMP-9, and TIMP-1 from the rats at the end of the experiment.

Group	MMP-2 (ng/mL)	MMP-9 (ng/mL)	TIMP-1 (ng/mL)
Normal control	2.65 ± 1.07	9.01 ± 2.34	1.42 ± 0.55
Cirrhosis control	8.43 ± 0.86**	45.61 ± 1.88**	6.09 ± 1.35**
Reference control	3.34 ± 0.13*	16.72 ± 2.43*	1.77 ± 0.06*
Low dose *B. rotunda *	5.86 ± 0.26	30.21 ± 4.43*	2.06 ± 0.19*
High dose *B. rotunda *	3.86 ± 0.69*	14.80 ± 2.30*	1.82 ± 0.05*

MMP-2: matrix metalloproteinase-2, MMP-9: matrix metalloproteinase-9, TIMP-1: metalloproteinase inhibitor-1. Data are expressed as mean ± SEM. Means among groups (*n* = 6 rats/group) show significant difference. *P < 0.05 compared to cirrhosis group. **P < 0.05 compared with normal group.
